The article "A Novel Immune-Associated Gene Signature for Overall Survival Prediction in Patients with Oral Squamous Cell Carcinoma" was retracted in 2023. Reasons: signs of a paper mill; compromised peer review; unreliable results or conclusions.

# A Novel Immune-Associated Gene Signature for Overall Survival Prediction in Patients with Oral Squamous Cell Carcinoma

**DOI:** 10.1155/2022/1063130

**Published:** 2022-04-13

**Authors:** Jian Yang, Zhien Feng, Xiaohong Yuan, Zhengxue Han

**Affiliations:** ^1^Department of Oral and Maxillofacial-Head and Neck Oncology, Beijing Stomatological Hospital, Capital Medical University, Beijing 100050, China; ^2^Department of Stomatology, Xinhua Hospital, Beijing 101100, China; ^3^Department of Oral Pathology, Beijing Stomatological Hospital, Capital Medical University, Beijing 100050, China

## Abstract

**Objective:**

To explore a novel Immune-associated gene signature for overall survival (OS) in patients with oral squamous cell carcinoma (OSCC).

**Methods:**

Expression profiles of genes and corresponding clinical materials of OSCC patients were obtained through the TCGA database. With a LASSO Cox regression model, a multigene signature was established to predict the OS of OSCC patients. Some molecular experiments including RNA interference, MTT, and Transwell assay were applied to verify the role of the risk gene FGF9 in OSCC.

**Results:**

43 immune-related prognostic DEGs were identified in OSCC. A 17-gene signature was established to assign the patients to either a high-risk group (HG) or a low-risk group (LG). The HG presented a shorter OS than the LG (*P* < 0.05). According to multivariate Cox regression analyses, the risk score was considered an independent factor for OS prediction (training set: HR = 3.485, 95% CI = 2.037–5.961, *P* < 0.001; test set: HR = 4.531, 95% CI = 2.120–9.682, *P* < 0.001). ROC curve-based analysis revealed the signature's ability for prediction. According to functional analysis, the immune cell expression and immune function of the HG were significantly inhibited. After knocking down the high-risk gene FGF9, the migration, proliferation, and invasion capabilities of OSCC cells HSC6 were significantly suppressed (*P* < 0.05).

**Conclusion:**

A novel immune-associated gene signature was identified for predicting the prognosis of OSCC. These risk genes show great potential as targets for OSCC treatment.

## 1. Introduction

Oral and maxillofacial malignancies include oral squamous cell carcinoma (OSCC), glandular epithelial carcinoma, and basal cell carcinoma, among which OSCC is the most common. According to reports, the incidence of OSCC ranks sixth in malignant tumors, and its treatment includes surgery, radiotherapy, and chemotherapy. Recurrence and metastasis are found in about 50% of OSCC cases within 3 years after therapy. There are more than 145,000 cases of death each year, with a 5-year survival of approximately 50% [1, 2].

The article "A Novel Immune-Associated Gene Signature for Overall Survival Prediction in Patients with Oral Squamous Cell Carcinoma" was retracted in 2023. Reasons: signs of a paper mill; compromised peer review; unreliable results or conclusions.

At present, the formulation of postoperative treatment protocols and prediction of OCSS treatment outcomes mainly rely on the tumor differentiation grading and preoperative TNM staging, which, however, are considered less satisfactory [3]. A growing body of evidence has verified the impact of the immune system and the immune cells in the tumor microenvironment on the recurrence and metastasis of OSCC [4]. Tumor-infiltrating cytotoxic T lymphocytes and natural killer cells eliminate tumor cells and limit tumor progression [5], whereas immunosuppressive cells, such as suppressor cells derived from myeloid, tumor-correlated macrophages, and regulatory T cells, inhibit the immune activity of T cells, contribute to immune escape of tumor cells, and promote tumor progression [6]. Studies have revealed a regulatory network of immune-related genes behind the infiltration of immune cells. Immune-related genes are now considered important targets for tumor treatment and prognosis prediction. Studies have found unique advantages of immune genes as cancer prognostic indicators, including ovarian cancer, liver cancer, and pancreatic cancer [7–9]. In addition, a study reported that an immune gene panel was able to predict the prognosis of OSCC, but its prediction sensitivity was low and lacked molecular level verification [10].

In the present research, immune-associated prognostic genes were screened out based on OSCC samples in The Cancer Genome Atlas (TCGA) database to establish an immune-associated gene set with higher sensitivity and specificity for forecasting the outcome of OSCC. Molecular biology methods were used to verify the role of the core genes in the gene set in OSCC.

## 2. Methods and Materials

The protocol was approved by the Ethics Committee of Beijing Stomatological Hospital, Capital Medical University (BSH39879).

### 2.1. Data Collection of TCGA-OSCC Cohort

Based on the TCGA website till March 31, 2021 (https://portal.gdc.cancer.gov/repository), the data about RNA sequence and corresponding clinical information of 413 samples were downloaded. The cohort covered 380 OSCC samples and 32 control ones. The expression profiles of genes were subjected to normalization by the scale method offered in the limma R package. Normalized read count values were applied. Due to the accessibility of TCGA to the public, our research was exempted from the ratification of local ethics committees. Our research followed the TCGA access policies and publication guidelines (Figure 1: the flow chart).

### 2.2. Identification of Infiltrating Immune Cells Prognostic Immune-Associated DEGs in the TCGA Cohort

R language CIBERSORT algorithm was applied to assess the expression and relationship of 22 immune cells in OSCC. The screening criteria of CIBERSORT analysis was *P* < 0.05 [11]. R limma package was applied for identifying the DEGs in OSCC. Univariate Cox analysis of overall survival (OS) was performed to identify the genes with prognostic values. *P* values were changed via BH correction. Then, the intersection of DEGs and the immune gene set were extracted from the Immport database (https://www.immport.org) to obtain immune-related DEGs in OSCC. With the STRING database (https://www.string-db.org), a PPI network was generated for the overlapping immune-related prognostic DEGs.

The article "A Novel Immune-Associated Gene Signature for Overall Survival Prediction in Patients with Oral Squamous Cell Carcinoma" was retracted in 2023. Reasons: signs of a paper mill; compromised peer review; unreliable results or conclusions.

### 2.3. Establishment and Confirmation of a Prognostic Immune Infiltration-Associated Gene Signature

To minimize the overfitting risk, a prognostic model was developed by LASSO-penalized Cox regression analysis [12]. Through the “glmnet” R package, the LASSO algorithm was employed for variable determination and shrinkage. The sample data were randomly assigned to a TG1 and a TG2 using the “Create Data Partition” algorithm. To identify genes associated with prognostic risk in OSCC, LASSO regression analysis was performed for data processing of the training and testing groups. These were applied for constructing a risk model via the “glment” package in R. The risk score of these 17 risk-related genes was calculated through the formula below:

(1) $$\begin{array}{c} \text{Riskscore}=\sum_{i=1}^{n}{\text{Coefi}}^{*}xi, \end{array}$$

where Coefi is the regression coefficient of the risk-related genes, and xi is its z-score transformed relative expression. The risk score of every gene was obtained by multiplying the coefficient by the expression of the gene. All sample data were assigned to high- and low-risk subgroups in accordance with the median risk score.

PCA was conducted through the “prcomp” function of the “stats” R package. With t-SNE, the distribution of different groups was identified by the “Rtsne” R package. To analyze the survival of every gene, the “surv_cutpoint” function of the “survminer” R package was used to define the optimal cut-off expression. The “survival ROC” R package was used to perform time‐dependent ROC curve-based analyses for assessing the significance of the gene signature in prediction.

### 2.4. Functional and Pathway Enrichment Analyses

The “clusterProfiler” R package was used for both GO and KEGG analyses on the basis of the DEGs between the high-risk group (HG) and low-risk group (LG). ^*∗*^*P* < 0.05 values were changed via the BH method. ssGSEA in the “gsva” R package was adopted to calculate the infiltrating score of 16 immune cells as well as the activity of 13 immune-associated pathways [12].

The article "A Novel Immune-Associated Gene Signature for Overall Survival Prediction in Patients with Oral Squamous Cell Carcinoma" was retracted in 2023. Reasons: signs of a paper mill; compromised peer review; unreliable results or conclusions.

### 2.5. Cell Culture and RNA Interference

The human OSCC cell strain HSC6 was acquired from the CCTCC (Wuhan, CN) and subjected to incubation (37°C, 5% CO_2_) in DMEM (Sigma-Aldrich; Merck KGaA) comprising 10% FBS (Gibco; Thermo Fisher Scientific, Inc.) and 100 U/ml penicillin/streptomycin (Beyotime Institute of Biotechnology). siRNAs were adopted to transfect the cells via Lipofectamine® RNAiMAX transfection reagent (Thermo Fisher Scientific, Inc., MA, the States). HSC6 cells (1 × 10^5^ cells) were placed in 6-well plates in complete DMEM, followed by overnight incubation (37°C). The siRNA lipoRNAiMAX mixture was then transferred to incubation wells comprising cells suspended in 800 *μ*l DMEM (cell density: about 30–40% (2 × 10^5^ cells)). The control siRNA and FGF9 siRNA (Thermo Fisher Scientific, Inc., Massachusetts, the States) were used at a concentration of 50 nM. After 6-h culture (37°C), the medium was changed to a fresh one (comprising FBS + penicillin/streptomycin), followed by 48-h continuous incubation (37°C) before later experimentation. HSC6 cells were assigned to four experimental groups: CG, HSC6 cells transfected with negative control siRNA or KD-FGF9 groups, HSC6 cells transfected with FGF9 siRNA group.

### 2.6. The Isolation of RNA and Quantitative Real-Time qPCR

The total RNA of HSC6 cells was acquired using the TRIzol reagent (Invitrogen, California, the States), and its quality was guaranteed via the agarose electrophoresis. The RNA was then reverse-transcribed to acquire the complementary DNA (cDNA) using a corresponding kit supplied by Invitrogen (California, the States). Subsequently, an SYBR Green PCR kit (Takara, Japan) was adopted to quantify the genes at an mRNA level. The relative miRNA was calculated using the 2−^∆∆Ct^ method, with GAPDH used for a reference. The primer sequences were as below: FGF9 (F: 5′-ATGGCTCCCTTAGGTGAAGTT-3′, R: 5′-CACTTAACAAAAC-3′), GADPH (F:5′- GGAGCGAGATCCCTCCAAAAT −3′, R: 5′- AGCGAGCATCCCCCAAAGTT-3′).

### 2.7. Western Blot

The total proteins of the cells were obtained using RIPA lysis buffer (Beyotime Biotechnology, Shanghai, CN), and one BCA assay kit (ThermoFisher Scientific, the States) was adopted for protein concentrations assay. The lysates were treated with 10% SDS-PAGE to separate target proteins based on their molecular weight, and the proteins were transferred to the PVDF films (Millipore, the States), followed by blocking in 5% defatted milk. The films were then treated with first antibodies against FGF9 (1 : 1000, Santa, CA, the States) and incubated overnight at 4°C, the GAPDH (1 : 1500, Cell Signaling Technology, Massachusetts, the States), and were then probed with the second antibody.

The article "A Novel Immune-Associated Gene Signature for Overall Survival Prediction in Patients with Oral Squamous Cell Carcinoma" was retracted in 2023. Reasons: signs of a paper mill; compromised peer review; unreliable results or conclusions.

### 2.8. MTT Assay

With the methods adopted previously, cell viability was tested. Totally, 20 *μ*l of MTT (5 mg/ml; Sigma-Aldrich) was supplemented after transfection or therapy, and a further 4-h culture was carried out, followed by supplementation of DMSO (200 *μ*l) for dissolving the formazan. OD values (490 nm) were then tested, and the relative cell viability was computed (the nontreated cell vitality (control): 100%.

### 2.9. Cell Migratory Evaluation through Wound Healing Assay

Before the cell wound healing assay, the cells were placed in 6-well plates (5 × 10^5^ cells/ml) till the formation of a monolayer. The scratch area was tested under one microscope (Olympus, Japan) at 0 and 24 h. Under the microscope, the distance of cells migrating to the scratch area was measured, followed by analysis using ImageJ (NIH, the States).

### 2.10. Cell Invasive Evaluation through Transwell Assay

The cells (5 × 10^5^) were placed on the upper side of Matrigel-coated polycarbonate Transwell filters. For the determination of invasion, the cells were subjected to suspension in a medium without serum, and a serum-contained medium was added to the lower compartment. The cells were treated with 2-h incubation (37°C). The noninvasive cells in the upper compartment were wiped off using cotton swabs. The invasive cells on the lower membrane were treated by 10-min immobilization with 100% methanol, air-drying, and dyeing through crystal violet solution (C0121, Beyotime), followed by counting under one microscope.

### 2.11. Statistical Analyses

The Student's *t*-test was applied for comparing genes between tumor tissues and corresponding nontumourous tissues in expression. A difference comparison of proportions was conducted using the Chi-squared test. The ssGSEA scores of immune cells or pathways were compared via the Mann–Whitney test with *P* values adjusted via the BH method between HG and LG. The intergroup comparison of OS was performed using Kaplan–Meier analysis based on the log-rank test. Independent predictors of OS were identified through univariate and multivariate Cox regression analyses. All statistical processing was conducted via R software (Version 3.5.3) or SPSS (Version 23.0). If not specified above, *P* < 0.05 denotes statistical significance, and each *P*value was two tailed. The data of western blot, qPCR, Transwell, and wound healing was evaluated with the Student's *t*-test.

## 3. Results

### 3.1. Infiltrating Immune Cells and Tumor Microenvironment in OSCC

In OSCC, there was an infiltration correlation between immune cells. For example, CD8T cells and CD4 memory T cells activated were both bound up with resting infiltration positively; NK cells activated and mast cells resting infiltration positively correlated. M0 macrophages and CD4 memory T cells activated, the infiltration of CD8T cells, and M1 macrophages negatively correlated (Figure 2(a)).

The article "A Novel Immune-Associated Gene Signature for Overall Survival Prediction in Patients with Oral Squamous Cell Carcinoma" was retracted in 2023. Reasons: signs of a paper mill; compromised peer review; unreliable results or conclusions.

### 3.2. Immune-Related Prognostic DEGs in OSCC

246 immune-related genes and 71 prognostic-associated genes in total were identified. By taking the intersection of the two, 43 immune-related prognostic DEGs in OSCC were identified (Figure 2(b)) 43 genes included 25 OSCC risk genes (TAC1, OSTN, STC1, etc) and 18 OSCC protective genes (IL10, IL17F, FAM3B, etc.). Dangerous genes meant that gene expression positively correlated with the patient's OS, and protective genes meant that gene expression negatively correlated with the patient's OS. PPI network analysis suggests that there was a close interaction among these genes. The coexpression network suggested that these genes were also closely related at the expression level. The expression heat map showed that 27 of the 43 genes were highly expressed in OSCC (VEFGA, IL1A, IL10, etc.), and 16 genes were significantly low expressed in OSCC (IL36A, OSTN, IL17F, etc.) (Figures 2(c)–2(e)).

### 3.3. Establishment of a Prognostic Model in the Training Set

With LASSO regression analysis, an OSCC prognostic risk model containing 17 genes was established according to the 43 genes previously obtained. The 17 genes were FGF9, OSTN, TAC1, DEFA3, NPY, AIMP1, MIF, AREG, HBEGF, MLN, FGF17, GNRH1, TXLNA, CTSG, CCL22, DEFB1, and SEMA3A. The patients were assigned to either HG (*n* = 95) or LG (*n* = 95) based on median cut-off in the training set. PCA and t-SNE analysis revealed the distribution of patients from different risk groups in 2 directions (Figures 3(a)–3(d)). In the training group (Figure 3(e)), the HG showed a lower OS than the LG (*P* < 0.05). ROC survival curve analysis revealed that in the training set, the AUC area of the model was 0.806, 0.749, and 0.799 in the first to the third year, respectively, suggesting the high specificity and sensitivity of the model (Figure 3(f)).

### 3.4. Confirmation of the 17-Gene Signature in the Test Set

Based on the median cut-off value in the test set, the patients were assigned to either an HG (*n* = 95) or an LG (*n* = 95). PCA and t-SNE analysis revealed the distribution of patients from different risk groups in 2 directions (Figures 4(a)–4(d)). The HG showed a lower OS than the LG in the test set (*P* < 0.001, Figure 4(e)). ROC survival curve analysis showed that in the test set, the AUC area of the model was 0.654, 0.669, and 0.696 in the first to three years, indicating that the model has high sensitivity and specificity (Figure 4(f)).

The article "A Novel Immune-Associated Gene Signature for Overall Survival Prediction in Patients with Oral Squamous Cell Carcinoma" was retracted in 2023. Reasons: signs of a paper mill; compromised peer review; unreliable results or conclusions.

### 3.5. Independent Prognostic Value of the 17-Gene Signature

Univariate and multivariate Cox regression analyses among the available variables were conducted for ascertaining whether the risk score was one independent factor for forecasting OS prognosis. In the former analysis, the risk score was markedly bound up with OS in the training set and test set (HR = 4.300, 95% CI = 2.371–7.798, *P* < 0.001; HR = 5.086, 95% CI = 2.431–10.641, *P* < 0.001, respectively) (Figures 5(a) and 5(c)). According to confirmation results, after correction for other confounding factors (age, gender, and duration of disease), the risk score is still one independent factor for forecasting OS in the latter analysis (training set: HR = 3.485, 95% CI = 2.037–5.961, *P* < 0.001; test set: HR = 4.531, 95% CI = 2.120–9.682, *P* < 0.001; Figures 5(b) and 5(d)).

### 3.6. Functional and Pathway Analyses in the Training and Test Sets

For illustrating the biological functions and pathways bound up with the risk score, the DEGs between HG and LG were applied for GO enrichment and KEGG pathway analyses. According to functional analysis, DEGs were primarily enriched in immune-associated GO terms in both the training and test sets, including immune response, humoral immune response, and B-cell-mediated immunity (*P* < 0.05, Figures 6(a) and 6(c)). According to KEGG analysis, DEGs are mainly enriched in immune-associated pathways in the training and test sets, including cell adhesion molecules, Th17 cell differentiation, cytokine-cytokine receptor interaction, chemokine signaling path, and Th1 and Th2 cell differentiation (*P* < 0.05, Figures 6(b) and 6(d)). To deeply investigate the association of the risk score with immune status, the enrichment scores of diverse immune cell subpopulations and associated functions or pathways were quantified using ssGSEA. Striking differences were found between the HG and LG in immune cell infiltration, and significantly less infiltration of 14 immune cells was found in the HG than the LG in the training and test sets, such as aDCs, B cells, CD8+T cells, and DCs (*P* < 0.05, Figures 7(a) and 7(c)) 10 immune-related functions in the HG were lower than the LG in the training and test sets, such as APC costimulation, CCR, APC coinhibition, check point, and HLA (*P* < 0.05, Figures 7(b) and 7(d)).

### 3.7. Effect of the Risk Gene FGF9 on OSCC Cell Line HSC6

PCR and western blot results showed that siRNA successfully knocked down the expression of FGF9 in HSC6 cells (*P* < 0.05, Figures 8(a) and 8(b)). The findings of MTT suggested that the proliferation activity of HSC6 cells in the KD-FGF9 group was suppressed in contrast to the CG (*P* < 0.05, Figure 8(c)). Wound healing results revealed a markedly lower migration ability of HSC6 cells in the KD-FGF9 group than in the CG (*P* < 0.05, Figure 8(d)). The results of the Transwell migration experiment revealed a lower migration ability of HSC6 cells in the KD-FGF9 group than in the CG. Transwell invasion results revealed a lower migration ability of HSC6 cells in the KD-FGF9 group than in the CG (*P* < 0.05, Figure 8(e)).

The article "A Novel Immune-Associated Gene Signature for Overall Survival Prediction in Patients with Oral Squamous Cell Carcinoma" was retracted in 2023. Reasons: signs of a paper mill; compromised peer review; unreliable results or conclusions.

## 4. Discussion

SCC is a prevalent pathological type of oral and maxillofacial tumor. The unique anatomical structure of the oral cavity leads to recurrence or invasive metastasis of oral squamous cell carcinoma after surgery [13]. In recent years, the biological cell research of the tumor immune microenvironment has become a research hotspot in tumor prognosis determination. Research has found a critical role of immune cells of the tumor microenvironment in tumorigenesis [14]. In the present study, there are complex interactions among 22 immune cells in the OSCC-associated immune microenvironment, the most significant of which is the positive regulation of CD8+ T cells with activated CD4+ memory T cells. There is a negative regulatory effect of activated CD4+ T cells with M0 macrophages. The findings are in agreement with the results acquired by Li et al. in the analysis of immune infiltration of bladder cancer [15]. This suggests that the two significantly infiltrated cells may inhibit the progression of OSCC through interaction, while the effect of M0 macrophages is the opposite.

Studies have found that there are some important genes behind the differences in immune infiltration in the tumor microenvironment that regulate immune cells. Herein, 43 immune-related prognostic genes were identified in OSCC, and a new prognostic prediction model containing 17 genes was developed. Research has revealed a valuable contribution of these genes to cancer. For example, Yang et al. found that MIF can drive the malignant progression of pancreatic cancer [16]. Zhang et al. found that MIF can promote the perineural infiltration of salivary adenoid cystic carcinoma [17]. Wang et al. found that AREG can regulate the epithelial-mesenchymal transition of pancreatic carcinoma cells [18]. Reddy et al. found that TAC1 is a cancer-promoting factor for breast cancer [19]. These results suggested that the dangerous genes may affect the malignant process of tumors, and their high expression may be associated with a worse prognosis in OSCC patients. Additionally, the protective genes in the new gene concentration have also been found to have important anticancer effects. It has been reported that CCL22 controls T-cell immunity by recruiting Tregs to tumor tissues and facilitating the formation of DC-Treg contacts in the lymph nodes [20]. Lv et al. found that the high expression of TXLNA indicates a good prognosis for pancreatic cancer [21]. These genes are an important guarantee for the gene set contributing to an accurate prognosis prediction of OSCC.

The article "A Novel Immune-Associated Gene Signature for Overall Survival Prediction in Patients with Oral Squamous Cell Carcinoma" was retracted in 2023. Reasons: signs of a paper mill; compromised peer review; unreliable results or conclusions.

In the present research, the new prediction model can accurately distinguish high- and low-risk OSCC patients, with high sensitivity and specificity. Therefore, the novel model shows great potential as an auxiliary prognostic prediction target. Moreover, in the analysis of independent risk factors, the tumor staging of OSCC is one of the independent risk factors, which is consistent with the nature and characteristics of malignant tumors [22]. Risk score, as one independent prognostic risk factor, outperforms tumor staging and grading in OSCC prediction. The findings of immune function analysis herein revealed that the tumor immune system of the HG was suppressed compared with the LG. Accordingly, immunotherapy can awaken the damaged immune system by rescuing depleted T cells and regulating immunosuppressive cells [23]. Compared with similar research [10], the model obtained here was based on a larger sample size and a larger AUC area, indicating higher sensitivity and specificity of the model. Furthermore, to further ascertain the accuracy of the model, the effect of the risk gene FGF9 in the model was verified by molecular biology. Studies have shown that FGF9 has an important cancer-promoting effect in gastric cancer and lung cancer [24, 25]. Nevertheless, the role of FGF9 in OSCC has not been reported. The present research confirmed that the propagation, migration, and invasiveness of OSCC cells were notably inhibited after FGF9 was knocked down. The results suggested that FGF9 was a risk factor for OSCC and confirmed the accuracy of the prediction model developed herein.

## 5. Conclusion

An OSCC prognosis prediction model was established based on immune genes with good prediction efficiency. The model risk genes show great potential as new targets for OSCC diagnosis and therapy and are worthy of in-depth study.

## Figures and Tables

**Figure 1:** Research strategy flow chart of this research.

**Figure 2:** Identification of immune-related prognostic genes in OSCC. (a) Expression and relationship of 22 immune cells in OSCC; (b) Venn diagram of 43 immune-related prognostic DEGs in OSCC; (c) forest plot of 43 immune-related prognostic DEGs in OSCC; (d) PPI network of the 43 genes; (e) coexpression network of the 43 genes.

**Figure 3:** Prognostic analysis of the 17-gene signature model in the training set. (a) The distribution and median value of the risk scores in the TCGA cohort. (b) PCA plot of the training set. (c) t-SNE analysis of the training set. (d) The distributions of OS status, OS and risk score in the training set. (e) Kaplan–Meier curves for the OS of patients in the HG and LG in the training set. (f) AUC of time-dependent ROC curves verified the prognostic performance of the risk score in the training set.

The article "A Novel Immune-Associated Gene Signature for Overall Survival Prediction in Patients with Oral Squamous Cell Carcinoma" was retracted in 2023. Reasons: signs of a paper mill; compromised peer review; unreliable results or conclusions.

**Figure 4:** Validation of the 17-gene signature in the test set. (a) The distribution and median value of the risk scores in the test set. (b) PCA plot of the test set. (c) t-SNE analysis of the test set. (d) The distributions of OS status, OS and risk score. (e) Kaplan–Meier curves for the OS of patients in the HG and LG. (f) AUC of time-dependent ROC curves in the test set.

**Figure 5:** The univariate and multivariate Cox regression analyses regarding OS in the training set (a, c) and the test set (b, d).

**Figure 6:** Function and pathway analyses of DEGs between the different risk groups in the training set (a, b) and the test set (c, d).

**Figure 7:** Comparison of the ssGSEA scores between different risk groups in the training set (a, b) and test set (c, d). The scores of 16 immune cells (a, c) and 13 immune-related functions (b, d) are displayed in boxplots. ns, not significant; ^*∗*^*P* < 0.05; ^*∗∗*^*P* < 0.01; ^*∗∗∗*^*P* < 0.001.

**Figure 8:** The effect of the risk gene FGF9 on OSCC cell line HSC6. PCR and western results showed that siRNA successfully knocked down the expression of FGF9 in HSC6 cells. (a–c). MTT assay revealed the proliferation ability of HSC6 cells in the KD-FGF9 group was significantly inhibited compared with the CG. (d) Wound healing assay revealed the migratory ability of HSC6 cells in the KD-FGF9 group was significantly lower than that of the CG. (e) Transwell assay revealed the migration and invasion ability of HSC6 cells in the KD-FGF9 group was obviously lower than that of the CG. ^*∗*^*P* < 0.05.

## Data Availability

The data sets used during the present study are available from the corresponding author upon reasonable request.
